# Analysis of Placement Priorities and Nursing Countermeasures of Transnasally Inserted Intestinal Obstruction Catheters in Patients with Acute Small Bowel Obstruction

**DOI:** 10.1155/2022/7317505

**Published:** 2022-09-29

**Authors:** Xiaoli Qian, Wei Yan

**Affiliations:** Department of General Surgery, General Hospital of Eastern Theater Command, Nanjing, Jiangsu 210001, China

## Abstract

**Objective:**

To explore the placement priorities and analysis of nursing countermeasures of transnasally inserted intestinal obstruction catheters in patients with acute small bowel obstruction (ASBO).

**Methods:**

One hundred and three patients with ASBO treated in our hospital from May 2016 to February 2022 were enrolled to this study. Patients who received individual nursing for transnasally inserted intestinal obstruction catheters were considered as the observation group (*n* = 59) and those who received traditional nursing were regarded as the control group (*n* = 44). The symptom relief time, daily gastrointestinal decompression, bowel sound recovery time, exhaust, defecation recovery time, and gas-liquid plane disappearance time were compared between both groups. The abdominal pain was evaluated by visual analogue scale (VAS), and the psychology of patients was evaluated by self-rating anxiety scale (SAS) and self-rating depression scale (SDS). Patients' clinical efficacy and incidence of adverse effects were counted, and quality of life was assessed using the short form 36 (SF-36) health survey questionnaire.

**Results:**

In the observation group, the improvement time of clinical symptoms and VAS, SAS, and SDS scores after intubation were lower than those of the control group, while the total clinical treatment efficiency was higher (*P* < 0.05). As to the adverse effects, the observation group was lower than the control group (*P* < 0.05). Also, the SF-36 scores were higher than those of the control group in all dimensions (*P* < 0.05).

**Conclusion:**

The individual nursing strategy implemented for the transnasally inserted intestinal obstruction catheter can effectively shorten the recovery of ASBO patients and improve their treatment outcome and prognosis quality of life.

## 1. Introduction

Acute small bowel obstruction (ASBO) is one of the familiar acute abdominal conditions in surgery, most of which have predisposing factors and a history of open surgical treatment [1]. The onset is marked by abdominal pain, bloating, nausea, vomiting, and cessation of anal discharge and defecation [2]. Besides, ASBO patients often have fluid and electrolyte loss, which can lead to necrosis and infection, and vomiting can be very frequent and the patients may even go into shock if no treatment is given [3]. At this stage, most clinical patients are treated with gastrointestinal decompression. The aim is to avoid infection, reduce edema of the bowel wall, relieve symptoms, and promote repair. The most common decompression method is to insert a gastric tube and use a negative pressure suction device to extract gastric juice, intestinal juice, and gas in the gastrointestinal tract, or using an enema to promote the excretion of intestinal contents through the anus can also reduce gastrointestinal pressure and achieve the purpose of reducing the symptoms of intestinal obstruction [4].

Transnasally inserted catheter therapy for intestinal obstruction is an important method to help decompress patients' stomachs and intestines by placing a catheter to effectively decompress the intestinal lumen above the site of obstruction [5]. The transnasally inserted intestinal obstruction catheter decompresses the site more deeply and more completely than the normal gastric tube decompression [6]. But the fixation method of the transnasally inserted intestinal obstruction catheter differs from that of the common gastrointestinal decompression tube, and the proper fixation of its position is relevant to the treatment outcome. So, the fixation point needs to be adjusted daily to prevent the catheter from going deeper or dislodging [7]. Furthermore, intestinal obstruction is prone to complicate ionic disturbances and acid-base imbalance and also to cause a variety of adverse effects [8]. Therefore, it is also vital to adopt nursing interventions along with treatment for early recovery of ASBO patients. However, the current clinical care content for ASBO is still lacking in specificity, and for the treatment of more complex transnasally inserted intestinal obstruction catheters, traditional nursing strategies are obviously not enough [9]. At present, many authors have pointed out that a targeted nursing strategy for ASBO and transnasally inserted intestinal obstruction catheters needs to be found as soon as possible in the clinic, but no significant results have been achieved so far [10, 11].

In this research, we analyzed the placement priorities and nursing countermeasures of transnasally inserted intestinal obstruction catheters in ASBO patients to provide valuable reference and guidance for future clinical management.

## 2. Materials and Methods

### 2.1. Study Area

The study was carried out at department of general surgery, General Hospital of Eastern Theater Command from May 2016 to May 2022.

### 2.2. Data Collection

One hundred and three patients with ASBO treated with transnasally inserted intestinal obstruction catheters in our hospital from May 2020 to February 2022 were regarded as the research objects. Inclusion criteria were as follows: (1) the diagnosis of ASBO is confirmed by imaging [12], and all patients reveal abdominal pain, abdominal distension, anal failure of stool and gas pass; (2) patients are older than 18 years; (3) complete case data; and (4) good compliance and no transfer. Exclusion criteria were as follows: (1) patients with intestinal obstruction caused by tumors; (2) patients without drug allergies; (3) patients with abnormal heart, liver, and kidney functions; and (4) pregnant and lactating women. Patients receiving individual nursing for the transnasally inserted intestinal obstruction catheter were considered the observation group (*n* = 59) and those receiving traditional nursing were regarded as the control group (*n* = 44). Included patients were informed about this trial and had signed an informed consent form.

### 2.3. Post-Admission Treatment

After admission, both groups were treated with fasting, anti-inflammatory, fluid replacement and maintenance of water-electrolyte balance, followed by treatment with a transnasally inserted intestinal obstruction catheter, all done by the same clinician in our hospital.

### 2.4. Nursing Strategies

After admission of patients in both groups, healthcare workers first established intravenous access, monitored vital signs, informed the treatment process, improved cooperation between family members and patients in treatment, helped patients eliminate adverse emotions, and made timely interventions for their needs. Since the patients in the observation group were treated with transnasally inserted intestinal obstruction catheters, due to the different fixation methods, the medical staff had to mark the catheters daily, observe and record the length of each patient's catheter outside the nasal cavity, make timely adjustments for deep or dislodged catheters, and promptly dump the drainage fluid to prevent catheter dislodgement. Patients also need to be advised to reduce large movements so as not to affect catheter twisting, etc. Furthermore, patients were closely observed daily for the occurrence of complications and timely communication with physicians, and successful cases were explained to patients and their families to enhance their confidence. The staff also give daily oral care to patients, keep the ward quiet, and create a good ward environment until they recover.

### 2.5. Outcome Measures

The improvement of clinical symptoms (time of symptom relief, average daily gastrointestinal decompression volume, time of recovery of bowel sounds, time of recovery of exhaustion and defecation, and time of disappearance of air-fluid plane) in both groups was observed and recorded. Abdominal pain after intubation was assessed via visual analogue scale (VAS) [13], and the psychology of patients was evaluated via self-rating anxiety scale (SAS) [14] and self-rating depression scale (SDS) [15]. The efficacy of both groups of patients was analyzed: markedly effective—patients' symptoms disappeared, and bowel movements and exhaustion returned to normal; effective—patients' symptoms disappeared, and the obstruction was dramatically improved; ineffective—the condition of patients did not improve or even worsen. Effective rate = (markedly effective + effective)/total number of cases × 100%). Complication rates were compared between both groups. The quality of life after treatment was assessed via the short form 36 (SF-36) health survey questionnaire [16].

### 2.6. Statistical Methods

The SPSS23.0 software was used for statistical analysis, and data were expressed as mean ± standard deviation and assessed via independent sample *t*-test. The count data were evaluated via the chi-square test, with *P* < 0.05 indicating a statistically remarkable difference.

## 3. Results

### 3.1. Summary of Results

In the observation group, the improvement time of clinical symptoms and VAS, SAS, and SDS scores after intubation were lower than those of the control group, while the total clinical treatment efficiency was higher, and the SF-36 scores were higher than those of the control group (*P* < 0.05).

### 3.2. Baseline Data of Two Groups of Patients

Baseline data such as age, gender, body mass index (BMI), type of obstruction, and ethnicity were statistically calculated for both groups, and there was no difference (*P* > 0.05), suggesting that both groups were experimentally comparable, as shown in Table 1.

### 3.3. Comparison of Improvement of Clinical Symptoms

The time to symptom relief in the observation group was (2.64 ± 1.17 d), which was dramatically shorter than that in the control group (*P* < 0.05, Figure 1(a)). In contrast, the average daily gastrointestinal decompression in the observation group was (729.27 ± 97.28 mL/d), which was higher than that in the control group (414.95 ± 66.29 mL/d) (*P* < 0.05, Figure 1(b)). The recovery time of bowel sounds was shorter in the observation group than in the control group (*P* < 0.05, Figure 1(c)). The recovery time of defecation and bowel movement in the observation group was clearly (3.89 ± 1.82 d) much lower than that in the control group (*P* < 0.05, Figure 1(d)). Finally, the disappearance time of the gas-liquid plane in the observation group was (9.66 ± 4.35 d), which was dramatically shorter than that in the control group (*P* < 0.05, Figure 1(e)).

### 3.4. VAS Score and Mentality Score after Intubation

The VAS score in the observation group was (3.27 ± 1.56), which was dramatically lower than that in the control group (5.70 ± 1.73) (*P* < 0.05, Figure 2(a)), indicating that the pain improvement in the observation group was better. Subsequently, the SAS and SDS scores of the observation group were (18.53 ± 3.06) and (16.85 ± 3.81), respectively, and both were lower than those of the control group (*P* < 0.05, Figures 2(b) and 2(c)), indicating that the post-treatment psychology of patients in the observation group was also better.

### 3.5. Comparison of Treatment Efficiency

The clinical efficacy of patients in both groups demonstrated that they were predominantly effective (52.5% in the observation group and 52.3% in the control group), but only 3.4% of patients in the observation group were ineffective, compared with 15.9% of those in the control group. The total efficacy rate of the observation group was 96.6%, which was higher than the rate of 84.1% in the control group (*P* < 0.05, Table 2).

### 3.6. Comparison of Incidence of Adverse Reactions

The incidence of adverse reactions during treatment in both groups was 5.1% in the observation group. Furthermore, nasopharyngeal discomfort occurred in 6.8% of patients in the control group, catheter dislodgement occurred in 4.5% of patients, electrolyte disturbance occurred in 4.5% of patients, and catheter blockage occurred in 4.5% of patients, for an overall adverse effect rate of 20.5%. The incidence of adverse reactions was lower in the observation group than in the control group (*P* < 0.05, Table 3).

### 3.7. Comparison of Quality of Life

To get a more comprehensive picture of patients' recovery, we assessed the quality of life of both groups. A PF score of (54.02 ± 7.05) was seen in the observation group, which was dramatically higher compared to the control group (*P* < 0.05, Figure 3(a)). The RP score in the observation group was (56.22 ± 5.14), which was likewise higher than that of the control group (*P* < 0.05, Figure 3(b)). BP scores were also higher in the observation group than in the control group (*P* < 0.05, Figure 3(c)). In addition, the GH score in the observation group was (84.78 ± 6.25), which was higher than the GH score in the control group (76.07 ± 6.91) (*P* < 0.05, Figure 3(d)). The VT score was higher in the observation group compared with the control group (80.85 ± 6.73 vs. 72.93 ± 7.08) (*P* < 0.05, Figure 3(e)). The SF scores of both groups were also higher in the observation group than in the control group (*P* < 0.05, Figure 3(f)). Similarly, the RE score in the observation group was (87.39 ± 5.99), which was higher than that in the control group (*P* < 0.05, Figure 3(g)). Finally, the MH scores in the observation group were higher (*P* < 0.05, Figure 3(h)).

## 4. Discussion

ASBO, as a highly prevalent emergency worldwide, is characterized by rapid onset and poor prognosis, and once the optimal treatment period is missed, it often endangers the life of patients [17]. The most basic treatment for ASBO is gastrointestinal decompression, but the nasogastric catheter is not long enough, which may lead to fluid and gas accumulation in the stomach and therefore affect the outcome of decompression [18]. To address this situation, a transnasally inserted intestinal obstruction catheter was prepared as an alternative in the clinical practice. However, with deeper catheter placement, patients will be at a much higher risk of adverse events such as impaired blood supply to the intestinal wall and wound infection [19]. Therefore, how to prevent the risk of adverse interventions more effectively in the application of transnasally inserted intestinal obstruction catheters has become a hot and difficult area of modern research.

In modern health care, there is a need not only for symptomatic treatment of patients' pathology but also for more appropriate care [20]. We have found that targeted nursing during invasive procedures such as prevention of mechanical ventilation infection and central venous placement via peripheral venipuncture can effectively reduce the probability of adverse patient events [21]. Therefore, this research will investigate targeted care strategies for the use of transnasally inserted intestinal obstruction catheters in ASBO treatment. It will provide an essential reference for nursing of transnasally inserted intestinal obstruction catheters for which reliable clinical guidance is currently lacking. As we mentioned above, the current clinical attention to transnasally inserted intestinal obstruction catheters is obviously insufficient, which directly leads to the unsatisfactory prognosis of ASBO patients [9]. Therefore, this study has very high guiding significance for ASBO patients treated with transnasally inserted intestinal obstruction catheters in the future. This may also be the key to preventing adverse complications of transnasally inserted intestinal obstruction catheters and improving clinical medical services in the future.

In this research, patients in the observation group had dramatically shorter clinical symptom improvement times than the control group after the implementation of nursing measures for the transnasally inserted intestinal obstruction catheter, indicating that the successful implementation of the nursing strategy adopted in this research can effectively improve the recovery of ASBO patients. Combining previous studies with our clinical experience, we summarized common problems in ASBO patients admitted to the hospital for transnasally inserted intestinal obstruction catheterization [22–26] and developed targeted nursing measures for these conditions.

*(1) Unhealthy Psychology*. When patients were first admitted to the hospital, their condition was serious. They had abdominal pain and distension, and they wanted to be relieved of their pain as soon as possible, with negative emotions of anxiety, tension, and fear. This research pointed out that maintaining an optimistic and good psychological state has a crucial significance in enhancing the treatment outcome of patients [27]. Thus, the nursing staff should observe the psychological changes of patients and explain the treatment plan, the procedure to be performed, the purpose of placing the intestinal obstruction catheter, the specific precautions to be taken after placement, and the safety and minimally invasive nature of placing the intestinal obstruction catheter and its good efficacy to make them confident by using scientific knowledge and easy-to-understand language. At the same time, the nursing staff also needs to pay attention to accompanying the family members' missionary work, and their encouragement and support will be a great comfort to patients, so that they can maintain an optimistic attitude to accept the treatment and increase the confidence to overcome the disease. In the end, the nursing staff should do a good job of catheter self-protection education according to patients' ability to accept, establish a good treatment atmosphere for them from various aspects and angles, and help them to establish confidence to overcome the disease.

*(2) Restricted Activity after Cannulation*. Due to the placement of the tube, the patient will lose the ability to move himself. This condition not only is detrimental to the recovery of the body's function but also may cause complications such as venous thrombosis and pressure sores in the lower extremities [28]. Hence, we will recommend patients to be more semi-recumbent at the time of placement and to get out of bed for 5–10 min with the assistance of family members if physical strength allows, which can greatly guarantee the active function of the body during the placement and promote functional recovery and resistance to adverse reactions.

*(3) Personal Nutrition and Diet Influence*. Due to the limited digestive function, patients' diet needs to be carried out in strict compliance with medical advice. If the intestinal obstruction is relieved and peristalsis returns to normal after treatment, patients can eat a liquid diet by mouth and then gradually transition to semi-liquid and general diet. The nursing staff arranged a reasonable infusion plan according to patients' dehydration and relevant blood biochemical indicators and closely observed the changes in condition and accurately recorded the in and out volume during the infusion. Patients are monitored regularly for liver and kidney function and electrolytes. Patients were also instructed to keep their mouths clean, to perform oral care three times a day, to remove nasal secretions in a timely manner, and to take nebulized inhalation treatment if they had throat discomfort.

*(4) Corresponding Treatment after Catheter Placement*. Due to the difference between the transnasally inserted intestinal obstruction catheter and the conventional nasogastric catheter, it does not need to be fixed at the nasal flank, and approximately 10–20 cm should be left between the nostril and the earlobe to allow the intestinal obstruction catheter to slide downward with intestinal peristalsis and prevent the catheter from twisting and folding. Meanwhile, patients and family members need to be reminded that they need to control their strength when performing turning to prevent the air bag from shifting or rupture. After the implementation of the above targeted measures, the VAS, SAS, and SDS scores and complication rates were lower in the observation group than in the control group, while the clinical outcomes were higher, which can fully verify the successful implementation of the nursing strategy. Furthermore, in a previous study, we saw that targeted individual nursing measures not only have excellent effects on improving patients' conditions but also further enhance their overall quality of life after treatment [29]. The quality of life of patients improves dramatically in the observation group, which is also due to the excellent effect of the implementation of the correct nursing strategy.

Of course, because there are no uniform guidelines for nursing of transnasally inserted intestinal obstruction catheters, the strategy implemented in this research may still have shortcomings that could be improved. We are not yet able to determine what the long-term prognosis of patients is due to the short experimental period. We will confirm the above limitations by conducting a sound experimental analysis as soon as possible.

## 5. Conclusion

The individual nursing strategy implemented for the transnasally inserted intestinal obstruction catheter can effectively shorten the recovery of ASBO patients and improve their treatment outcome and prognosis quality of life, which is worth promoting in the clinical setting.

## Figures and Tables

**Figure 1:** Comparison of improvement of clinical symptoms. (a) Comparison of time of symptom relief. (b) Comparison of average daily gastrointestinal decompression volume. (c) Comparison of time of recovery of bowel sounds. (d) Comparison of time of recovery of exhaustion and defecation. (e) Comparison of time of disappearance of air-fluid plane. Note: ∗ means *P* < 0.05 for the comparison between the two groups.

**Figure 2:** VAS score and mentality score after intubation. (a) Comparison of VAS scores. (b) Comparison of SAS scores. (c) Comparison of SDS scores. Note: ∗ means *P* < 0.05 for the comparison between the two groups.

**Figure 3:** Comparison of SF-36 score. (a) Comparison of the PF scores. (b) Comparison of the RP scores. (c) Comparison of the BP scores. (d) Comparison of the GH scores. (e) Comparison of VT scores. (f) Comparison of SF scores. (g) Comparison of RE scores. (h) Comparison of MH scores. Note: ∗ means *P* < 0.05 for the comparison between the two groups.

**Table 1:** Baseline data of two groups of patients.

	*N*	Age	Gender (male/female)	BMI (kg/m^2^)	Type of intestinal obstruction (complete/strangulated/incomplete)	Nationality (Han/minority)
Observation group	59	45.4 ± 1.7	31 (52.5)/28 (47.5)	27.0 ± 2.1	19 (32.2)/20 (33.9)/20 (33.9)	53 (89.8)/6 (10.2)
Control group	44	45.8 ± 1.4	24 (54.5)/20 (45.5)	26.1 ± 2.6	16 (27.1)/17 (28.8)/11 (18.6)	41 (93.2)/3 (6.8)
*χ* ^2^/*t*		1.302	0.041	1.942	0.949	0.355
*P*		1.196	0.840	0.055	0.622	0.551

**Table 2:** Comparison of treatment efficiency.

	*n*	Markedly effective	Efficient	Invalid	Total effective rate
Observation group	59	26 (44.1)	31 (52.5)	2 (3.4)	96.6%
Control group	44	14 (31.8)	23 (52.3)	7 (15.9)	84.1%
*χ* ^2^					4.954
*P*					0.026

**Table 3:** Comparison of incidence of adverse reactions.

	*n*	Nasopharyngeal discomfort	Catheter dislodgement	Electrolyte disturbance	Catheter blockage	Overall adverse effect rate
Observation group	59	1 (1.7)	1 (1.7)	1 (1.7)	0 (0.0)	5.1%
Control group	44	3 (6.8)	2 (4.5)	2 (4.5)	2 (4.5)	20.5%
*χ* ^2^						5.784
*P*						0.016

## Data Availability

The data used to support the findings of this study are available from the corresponding author upon request.
